The article "Interlaminar stabilization offers greater biomechanical advantage compared to interspinous stabilization after lumbar decompression: a finite element analysis" was published in 2020. Journal: J Orthop Surg Res.

# Interlaminar stabilization offers greater biomechanical advantage compared to interspinous stabilization after lumbar decompression: a finite element analysis

**DOI:** 10.1186/s13018-020-01812-5

**Published:** 2020-07-29

**Authors:** Teng Lu, Yi Lu

**Affiliations:** 1 Department of Neurosurgery, Brigham and Women’s Hospital, Harvard Medical School, 60 Fenwood Rd, BTM 4th floor, Boston, MA 02115 USA; 2 Department of Orthopedics, Xi’an Jiaotong University Second Affiliated Hospital, Xi’an, China

**Keywords:** Lumbar spinal stenosis, Finite element, Biomechanics, Surgical decompression, Fusion, Interlaminar stabilization, Interspinous stabilization, Coflex device, Complication

## Abstract

**Background:**

Interlaminar stabilization and interspinous stabilization are two newer minimally invasive methods for lumbar spine stabilization, used frequently in conjunction with lumbar decompression to treat lumbar stenosis. The two methods share certain similarities, therefore, frequently being categorized together. However, the two methods offer distinct biomechanical properties, which affect their respective effectiveness and surgical success.

**Objective:**

To compare the biomechanical characteristics of interlaminar stabilization after lumbar decompression (ILS) and interspinous stabilization after lumbar decompression (ISS). For comparison, lumbar decompression alone (DA) and decompression with instrumented fusion (DF) were also included in the biomechanical analysis.

**Methods:**

Four finite element models were constructed, i.e., DA, DF, ISS, and ILS. To minimize device influence and focus on the biomechanical properties of different methods, Coflex device as a model system was placed at different position for the comparison of ISS and ILS. The range of motion (ROM) and disc stress peak at the surgical and adjacent levels were compared among the four surgical constructs. The stress peak of the spinous process, whole device, and device wing was compared between ISS and ILS.

**Results:**

Compared with DA, the ROM and disc stress at the surgical level in ILS or ISS were much lower in extension. The ROM and disc stress at the surgical level in ILS were 1.27° and 0.36 MPa, respectively, and in ISS 1.51°and 0.55 MPa, respectively in extension. This is compared with 4.71° and 1.44 MPa, respectively in DA. ILS (2.06–4.85° and 0.37–0.98 MPa, respectively) or ISS (2.07–4.78° and 0.37–0.98 MPa, respectively) also induced much lower ROM and disc stress at the adjacent levels compared with DF (2.50–7.20° and 0.37–1.20 MPa, respectively). ILS further reduced the ROM and disc stress at the surgical level by 8% and 25%, respectively, compared to ISS. The stress peak of the spinous process in ILS was significantly lower than that in ISS (13.93–101 MPa vs. 31.08–172.5 MPa). In rotation, ILS yielded a much lower stress peak in the instrumentation wing than ISS (128.7 MPa vs. 222.1 MPa).

**Conclusion:**

ILS and ISS partly address the issues of segmental instability in DA and hypermobility and overload at the adjacent levels in DF. ILS achieves greater segmental stability and results in a lower disc stress, compared to ISS. In addition, ILS reduces the risk of spinous process fracture and device failure.

## Background

Surgical decompression with instrumented fusion (DF) has been commonly used to treat lumbar spinal stenosis (LSS), especially when it is associated with potential instability or deformity [1, 2]. Compared with decompression alone (DA), the additional instrumented fusion procedure enhances the stability and reduces the incidence of iatrogenic instability and secondary stenosis at the surgical level [3, 4]. However, it is also associated with the risk of pseudarthrosis, nonunion, instrumentation failure, and adjacent segment disease [3–5]. In recent decades, interlaminar or interspinous stabilization has been introduced as an alternative to DA or DF, either as a stand-alone device or in conjunction with decompression. Biomechanically, these techniques partly simulate the kinematics of the surgical level and provide segmental stability in extension [6, 7]. Until now, many interspinous stabilizing devices have been used for the treatment of LSS, such as X-STOP (Medtronic, MN, USA), WALLIS (Abbott Spine, TX, USA), and Superion (VertiFlex, San Clemente, CA, USA) [8–10]. Since first introduced in 1994, Coflex (Paradigm Spine, NY, USA) device, an interlaminar stabilization device, has been gaining popularity in clinical use [11–15]. Some studies have reported that decompression with Coflex stabilization achieves better outcomes than DA or DF, including a higher clinical success rate [12, 14, 15], more physiological kinematics [11, 12], a larger foraminal and disc height [11, 14, 15], and less influence on adjacent segments [13].

Despite these merits, interspinous or interlaminar stabilization devices can induce some novel complications that are unique to this surgical procedure, such as spinous process fracture, device breakage, and dislodgment [8, 9, 16]. Regarding the Coflex device, the incidence of device-related complications has been reported in up to 24.4% of these patients [17]. In some severe cases, an additional fusion procedure is required to relieve the symptoms [17, 18]. Excessive decompression, nonstandard operation, and osteoporosis have been considered causes of these complications [17–19]. Some studies have indicated that comparing with interlaminar positioning of the Coflex device, interspinous positioning might result in a greater stress load on the spinous process and therefore increase the incidence of device-related complications [17, 20], which implies that the interlaminar stabilization may be superior to the interspinous stabilization in the aspect of biomechanical performance. To the best of our knowledge, there is still a lack of biomechanical data to support this view and explain the mechanism.

Traditionally, the interlaminar devices and interspinous process devices are frequently categorized together [8, 21, 22]. Most previous studies have focused only on comparing interlaminar or interspinous device to other lumbar surgical techniques [9, 10, 12, 15, 23], and few studies have focused on assessing whether the position of such device placement has an influence on biomechanical or clinical outcomes. In order to assess whether there is a fundamental difference in the biomechanical performance of the interlaminar device and interspinous process device, we comprehensively compared the biomechanical characteristics of DA, DF, decompression with interlaminar stabilization (ILS), and decompression with interspinous stabilization (ISS) by using the finite element (FE) methods. To minimize the specific device influence on the biomechanical evaluation, we used Coflex as a model system for the ILS and ISS comparison.

## Methods

### Finite element (FE) modeling of the lumbar spine

A nonlinear FE model of the L2–L5 lumbar spine was constructed (Fig. 1a). To create this model, thin layer (0.625 mm) computed tomography images (SOMATOM Definition Flash, Siemens, Inc., Muenchen, Germany) of the L2–L5 lumbar spine of a young healthy male were converted to a surface model using a medical image-based engineering software (Mimics, Materialise, Inc., Leuven, Belgium). Solid models of the cortical shell, cancellous bone, and intervertebral discs were constructed using 3-Matic (Materialise, Inc., Leuven, Belgium). HyperMesh (Altair Engineering, Inc., Troy, MI, USA) was used for model meshing, and Abaqus (Hibbitt, Karlsson and Sorenson, Inc., Providence, RI, USA) was used for material property definition, model assembly, and FE analysis.

**Fig. 1:** FE models of **a** intact L2–5 lumbar spine, **b** DA, **c** DF, and **d** ILS and **e** ISS

The thickness of the cortical shell and cartilage endplate was set as 1 mm and 0.5 mm, respectively [24, 25]. The volume of the nucleus pulposus accounted for approximately 35% of the intact intervertebral disc [26]. The annulus fibrosus was modeled as a combination of annulus ground substance and annulus fibers. Eight layers of annulus fibers were defined as truss elements and embedded into the ground substance at an inclination of ± 25–35° [26, 27]. The elastic strength of the annulus fibers proportionally decreased from the outermost layer (550 MPa) to the innermost (360 MPa) layer [27, 28]. The ligaments constructed in the FE model were defined as truss elements that respond nonlinearly in tension only [27, 28]. Frictionless soft-contact between the articular processes was applied to mimic articular cartilage [29]. The bony tissues, nucleus pulposus, and the implants were modeled as elastic elements. The elements of the annulus ground substance were defined as hyperelastic. And hypoelastic material properties were assigned to the ligaments and annulus fibers. A convergence analysis was performed by ensuring the maximum changes in the strain energy < 5%. The element types and the material properties used in this FE model were assigned based on previous publications, which are shown in Table 1 [27, 28].

**Table 1:** Material properties assigned to the FE model

Component	Element type	Young modulus (MPa)	Poisson ratio	Cross-sectional area (mm^2^)
Bone				
Cortical bone	C3D4	12,000	0.3	
Cancellous bone	C3D4	100	0.2	
Cartilage endplate	C3D8	24	0.4	
Intervertebral disc				
Nucleus pulpous	C3D8	1	0.49	
Annulus ground substance	C3D8H	Hyperelastic (C10 = 0.18, C01 = 0.045)		
Annulus fibers	T3D2	Hypoelastic (360–550 MPa)		
Ligaments				
Anterior longitudinal	T3D2	15.6 (< 12%), 20 (> 12%)		63.7
Posterior longitudinal	T3D2	10 (< 11%), 20 (> 11%)		20
Ligamentum flavum	T3D2	15 (< 6.2%), 19.5 (> 6.2%)		40
Capsular	T3D2	7.5 (< 25%), 32.9 (> 25%)		30
Interspinous	T3D2	10 (< 20%), 11.6 (> 20%)		40
Supraspinous	T3D2	8.0 (< 20%), 15 (> 20%)		30
Intertransverse	T3D2	10 (< 18%), 58.7 (> 18%)		2
Implants				
Coflex device, screws, and rods (titanium)	C3D4	110,000	0.3	

### FE modeling of the surgical procedures

In total, four surgical constructs were modeled and compared in this study, i.e., DA, DF, ILS, and ISS. Using Coflex device as a model, ILS and ISS models were constructed. For the surgical model of DA, bilateral decompression at L3/4 was simulated by removing the supraspinous ligament, interspinous ligament, ligamentum flavum, part of the laminar, and 50% of the medial facet (Fig. 1b) [7]. For the surgical model of DF, a screw-rod fixation system was added at the surgical level after decompression (Fig. 1c). The diameter and length of the screw was 6.5 mm and 45 mm, respectively. The diameter of the rod was 5.5 mm. A “tie” constraint was assigned to the screw-rod and screw-bone interfaces to simulate the conditions of rigid fixation.

The geometry of the Coflex device was constructed based on the real product. A device with a suitable height (10 mm) was chosen and inserted into the interlaminar or interspinous space. Part of the spinous process was removed to provide sufficient space for Coflex implantation. The surface between the Coflex device and the bony tissues was defined as surface-to-surface contact. The coefficient of friction in the region where the wing contacted the spinous process was set to 0.8. A much lower coefficient of friction (0.1) was set for the rest of the contact region [7]. The ILS and ISS constructs were modeled by inserting the Coflex device into the interlaminar or interspinous space (Fig. 1d–e). For the surgical construct of ILS, the anterior portion of the Coflex device was located in the interlaminar space of the decompression level (Fig. 2a). In comparison, in the surgical construct of ISS, the whole “U” structure of the Coflex device was located in the interspinous space (Fig. 2b).

**Fig. 2:** **a** In ILS, the anterior portion of the Coflex device was inserted into the interlaminar space. **b** In ISS, the entire Coflex device was inserted into the interspinous space

### Loading conditions

For all the FE models, the interior surface of L5 was constrained. A compressive load of 400 N was imposed on the superior surface of L2 to simulate physiological compressive loading [30]. For the intact FE model, another 8 Nm was applied to L2 to simulate flexion, extension, bending, and axial rotation [30]. For validation of the intact L2–L5 FE model, the segmental ROMs (L2/3, L3/4, and L4/5) were compared with the outcomes of previous biomechanical and FE publications [7, 30, 31]. For the surgical models, a hybrid method was applied, in which specific moments were applied to produce the same total ROMs of the intact FE model [7, 32].

## Results

### Model validation

The intersegmental ROMs of the intact FE model are listed in Table 2. The results are in accordance with those of previous publications (Fig. 3), suggesting that the intact L2-L5 FE model in the present study was successfully constructed and could be used for further modeling and analysis.

**Table 2:** Intersegmental ROM and disc stress peak of the FE models

	Intersegmental ROM (°)			Disc stress peak (MPa)		
	L2/3	L3/4 (surgical segment)	L4/5	L2/3	L3/4 (surgical segment)	L4/5
Extension						
Intact	2.68	2.88	3.75	0.73	0.78	0.72
DA	1.91	4.71	2.99	0.69	1.44	0.74
DF	3.86	0.41	5.35	0.89	0.06	0.82
ILS	3.49	1.27	4.85	0.84	0.36	0.80
ISS	3.42	1.51	4.78	0.83	0.55	0.80
Flexion						
Intact	3.92	4.42	5.31	0.76	0.70	0.76
DA	3.27	5.68	4.69	0.66	0.76	0.65
DF	5.24	1.12	7.20	0.88	0.57	0.88
ILS	3.31	5.64	4.75	0.67	0.75	0.66
ISS	3.27	5.65	4.69	0.66	0.75	0.65
Bending						
Intact	3.17	3.21	3.78	0.82	1.05	0.97
DA	3.04	3.30	3.81	0.81	1.18	0.96
DF	4.12	0.99	5.05	0.98	0.50	1.20
ILS	3.12	3.12	3.92	0.83	1.08	0.98
ISS	3.12	3.12	3.92	0.83	1.08	0.98
Rotation						
Intact	1.94	2.10	2.15	0.36	0.45	0.43
DA	1.98	2.14	2.07	0.37	0.45	0.41
DF	2.50	0.95	2.74	0.37	0.36	0.47
ILS	2.06	1.99	2.14	0.37	0.48	0.42
ISS	2.07	1.98	2.15	0.37	0.49	0.42

*ROM* range of motion, *DA* decompression alone, *DF* decompression with fusion, *ILS* decompression with interlaminar stabilization, *ISS* decompression with interspinous stabilization

**Fig. 3:** Comparison of the intersegmental ROM between the current intact model and the outcomes of previous publications

### Intersegmental ROM and disc stress peak

The resulting intersegmental ROM and disc stress peak are shown in Table 2. Figure 4 shows the results that were normalized with respect to the intact model.

**Fig. 4:** Comparison of the normalized intersegmental range of motion (ROM) and disc stress peak among the intact, DA, DF, ILS, and ISS models

For the surgical segment (L3/4), the DF procedure resulted in the lowest ROM and disc stress peak in the four physiological motions. Compared with the intact model, the DF model showed values decreased by 69–86% and 52–94%, respectively. For the DA model, the ROM and disc stress peak did not change obviously in bending or rotation. However, in extension and flexion, the ROM increased by 63% and 29%, respectively, and the disc stress peak increased by 85% and 9%, respectively. The ROM and disc stress peak in bending and rotation in the ILS and ISS models were similar to those in the intact model. In extension, ISS reduced the ROM and disc stress peak by 48% and 29%, respectively. Compared with ISS, ILS further decreased the ROM and disc stress peak by 8% and 25%, respectively. In flexion, in both ILS and ISS model, the ROM and disc stress peak increased similarly by 28% and 7%, respectively.

In the adjacent segments (L2/3 and L4/5), the DF model yielded the highest ROM and disc stress peak in the four motions. Compared with the intact model, the DF model showed ROM and disc stress peak values at the adjacent segments increased by 27–44% and 3–24%, respectively. For the DA model, the ROM and disc stress peak did not change obviously in bending or rotation. However, in extension and flexion, the ROM and disc stress peak at the adjacent segments were reduced by 12 to 29% and − 3 to 12%, respectively. The ROM and disc stress peak in bending and rotation in the ILS and ISS models were similar to those in the intact model. In flexion, the two surgical models reduced the ROM and disc stress peak at the adjacent segments by 11–17% and 11–14%, respectively. In extension, the ROM and disc stress peak at the adjacent segments were increased by 27–30% and 11–15%, respectively.

### Stress peak of the spinous process and Coflex device

Figure 5 shows the stress peak of the spinous process and Coflex device in the surgical constructs. The stress peak of the L3 spinous process was 13.93–71.02 MPa in ILS, which was much lower than that in ISS (34.57–159.9 MPa), especially in extension and rotation. The stress peak of the L4 spinous process was 25.4–101 MPa in ILS, which was also lower than that in ISS (31.08–172.5 MPa), especially in extension. The stress distributions of the L3 and L4 spinous processes are shown in Fig. 6.

**Fig. 5:** Comparison of the stress peak of the spinous process, whole Coflex device, and Coflex wing between ILS and ISS

**Fig. 6:** Stress distributions in the L3 and L4 spinous processes

The stress peak of the intact Coflex device was similar in ILS and ISS (19.63–207.7 MPa vs. 16.75–222.1 MPa). The stress peak of the Coflex wings in ILS and ISS was 19.63–212.7 MPa and 16.75–222.1 MPa, respectively. The highest stress peak was found in the ISS model in rotation (222.1 MPa), which was increased by 73% compared with that in the ILS model (128.7 MPa). The stress distributions of the Coflex devices are shown in Fig. 7.

**Fig. 7:** Stress distributions in the Coflex device

## Discussion

In 1986, the first interspinous device named WALLIS was introduced [8]. After that, many interlaminar or interspinous devices have been developed [8, 33]. The aim of using these devices in conjunction with lumbar decompression surgery is to enhance the stability after alleviating the nerve compression at the surgical level [8, 22, 33]. Due to the similar design theories, the interlaminar devices and the interspinous devices are commonly classified into one category [8, 21, 22]. However, the placing positions of the two types of device are much different. The interlaminar devices were designed to be inserted into the interlaminar space whereas the interspinous devices were placed between the adjacent spinous processes. Until now, few studies have attempted to assess the biomechanical difference between the two surgical constructs.

In the current FE study, we comprehensively compared the biomechanical characteristics of ILS and ISS to evaluate whether ILS is superior to ISS in terms of biomechanical performance. During the modeling procedure, we used the same Coflex device at different position for the modeling of the ILS and ISS constructs to minimize the influence of the device design on the biomechanical evaluation but to focusing on the effect of the device location. The reason for choosing the Coflex device was that this implant could be inserted into both the interlaminar and interspinous spaces [8]. In addition, the Coflex device is one of the commonly used interlaminar or interspinous devices in surgeries [11–13]. Our results suggested that the interlaminar device and interspinous device have different biomechanical properties and should not be simply categorized together. Compared with ISS, ILS significantly reduces the stress level on the spinous process and also significantly reduces the stress on the hardware itself during spine rotation. In addition, ILS further significantly reduces the disc stress compared to ISS placement at the surgical level.

As shown in the results, both the ILS and ISS procedures provided the surgical level with stability in extension by reducing the segmental ROM and disc stress. Additionally, both surgical procedures effectively preserved the mobility of the surgical and adjacent levels in bending and rotation, compared to either DA or DF. The intersegmental ROM and disc stress peak were similar to those of the intact lumbar spine. However, in flexion, hypermobility and overload were observed at the surgical level, suggesting that the Coflex device could not provide strong biomechanical stability during flexion. This is mainly because the Coflex wings were crimped only to the spinous processes, and the effects of motion restriction in flexion are weak [6]. These results are in accordance with those of previous studies. Kulduk et al. conducted an FE study to assess the biomechanical performance of interlaminar device and found that the ROM at the surgical level was increased by 19% in flexion compared with that of the intact model [34]. Another FE study conducted by Lo et al. showed that the ROM and disc stress in the Coflex model were similar to those in the intact model in bending and rotation but much higher in flexion and lower in extension [7]. They concluded that Coflex device could effectively maintain the stability of the surgical level except in flexion [7]. Additionally, compared with the DF procedure, Coflex device has less biomechanical influence on the adjacent levels [7], which subsequently reduces the risk of adjacent segment degeneration [7, 12].

Compared with ISS, ILS further reduced the ROM and disc stress peak at the surgical level by 8% and 25%, respectively, suggesting that the ILS procedure has a greater capacity to maintain the stability of the surgical level. The reason for this phenomenon may be that the interlaminar position of the Coflex device is closer to the rotational center of the surgical segment [35, 35]. In flexion-extension, the rotational center of each segment has been reported to be mainly located in the posterior portion of the anterior column. Liu et al. used dual fluoroscopic imaging to measure the rotational center of L4/5 and L5/S1 in young adults [36]. The results showed that the rotational center in flexion-extension was located in the posterior quarter of the disc at L4/5 and near the posterior rim of the disc at L5/S1 [36]. A similar radiological study conducted by Aiyangar et al. showed that the average rotational center of each lumbar segment was located near the middle and posterior portions of the superior endplate [35]. Therefore, as the surgical segment extends, the ILS construct restricts the motion at an earlier stage because it is placed in the interlaminar space and thus closer to the rotational center. Meanwhile, a lower ROM in extension accordingly reduces the disc stress at the surgical level, which further decreased the risk of secondary degeneration [7, 12].

In addition, the ILS construct yielded much lower stress on the spinous process. In all motion directions, the average stress peak in the L3 and L4 spinous processes in the ISS construct was 96.15 MPa, which was approximately 1.75 times as high as that in the ILS construct (54.8 MPa). The reason for these results may be that the load in the posterior column was mainly transferred onto the laminar in the ILS construct [20]. As shown in the stress nephogram of the posterior column (Fig. 6), the stress peak in the ILS construct was mainly located on the laminar facet, whereas the stress peak in the ISS construct was on the spinous process. Compared with the spinous process, the laminar facet has a much greater stiffness and mechanical strength [20, 37]. A previous biomechanical study has reported that the laminar facet has a failure strength approximately five times higher than that of the spinous process (1966 N vs. 405 N), and thus has a greater capacity to resist fracture [37]. Additionally, the laminar facet offers a greater contact area for the Coflex device due to its wider dimension. Due to these advantages, the ILS construct results in a more homogeneous stress distribution in the posterior column and thus carries less risk of inducing spinous process fracture than the ISS construct [20, 38].

Regarding the stress peak of the Coflex device, the value was similar in ILS and ISS. However, for the wing structure, ISS yielded a much higher stress peak in rotation than did ILS (222.1 MPa vs. 128.7 MPa). The reason for this phenomenon may also be that the Coflex device in the ISS construct is farther away from the rotational center of the surgical segment [35, 36]. Since the ROM was similar in ILS and ISS in rotation, the ISS construct resulted in larger deformation of the wing structures and subsequently a greater stress load to resist segmental motion. In addition, due to the design features, the Coflex wing has much less fatigue strength than the Coflex U arm [20]. All of these disadvantages result in ISS increasing the risk of Coflex wing breakage; thus, the Coflex device should be inserted into the interlaminar space to avoid high stress concentration on the wings.

For the DA and DF procedures, the results of the current study showed that they significantly changed the biomechanical characteristics of the lumbar spine, which is in accordance with the findings of previous studies [7, 39]. Lo et al. performed an FE study to assess the biomechanical performance of different fusion techniques in treating lumbar spinal stenosis and found that the conventional fusion procedure increased the ROM at the adjacent levels by 21–44% in all motion directions [39]. For the DA procedure, another FE study conducted by Lo et al. showed that the ROM at the surgical level was increased by 13% and 64% in flexion and extension, respectively [7]. Meanwhile, in the same motion directions, the disc stress peak at the surgical level was 10% and 100% greater than that in the intact model in flexion and extension, respectively [7].

Our results showed that the use of ILS or ISS partly addresses the issue of segmental instability in the DA model. Both the two surgical procedures enhance the stability and reduce the load on the anterior column at the surgical level in extension, especially in ILS. These advantages may facilitate the achievement of better clinical outcomes in treating lumbar spinal stenosis. Schmidt et al. reported the clinical outcomes of DA and ILS in treating symptomatic lumbar spinal stenosis after 2 years [15]. The results showed that the clinical success rate was much higher in the ILS group (58.4% vs. 41.7%) [15]. A similar study conducted by Kumar et al. also showed that patients treated with ILS showed greater recovery of symptoms than those treated with decompression alone [14]. In addition, due to the strong support in the posterior column, the foraminal and disc height in the group treated with ILS were well maintained [14].

Meanwhile, ILS or ISS alleviated the hypermobility and overload at the adjacent levels compared with DF, which might subsequently reduce the risk of adjacent segment degeneration [7, 12]. In an FE study conducted by Shen et al., the results showed that DF significantly increased the ROM at the adjacent levels by 17.7–61.4%, which was much higher than those in ILS and ISS [22]. In addition, DF yielded much higher disc stress and facet joint stress at the adjacent levels than ILS and ISS [22]. Bae et al. retrospectively compared the clinical outcomes of using ILS and DF for treating lumbar spinal stenosis [12]. The results showed that the rate of composite clinical success at the treated level was similar in the ILS and DF groups (64.5% vs. 69.7%) and that both surgical procedures could provide sufficient stability at the treated level [12]. However, at the adjacent level, the DF procedure increased the angular motion by a mean of 1.42°, whereas the ILS procedure effectively maintained the normal kinematics [12]. The author considered that the more physiological mobility at the adjacent level could prevent segmental degeneration in ILS patients [12].

There exist some limitations in this study. First, the intact FE model was construct based on the computed tomography data from a young healthy man, which might underestimate the influence of severe degenerative pathologies on the biomechanical performance of the lumbar spine, such as severe osteoporosis, scoliosis, and significant losses of the disc height and segment lordosis. In addition, some other interlaminar and interspinous devices could be compared in the future to further understand the difference of the biomechanical properties between ILS and ISS.

## Conclusion

The ILS or ISS construct preserves better the biomechanical characteristics of the intact lumbar spine compared to the DA and DF constructs and partly addresses the issues of the DA construct in segmental instability and the DF construct in hypermobility and overload at the adjacent levels. Compared to the ISS construct, the ILS construct reduces the stress on the spinous process and on the device itself, potentially minimizing the possible complications. In addition, the ILS construct further reduces the disc stress or excessive range of motion at the surgical level, providing a greater capacity to maintain the natural integrity of the operated spine.

## Data Availability

All data generated or analyzed during this study are included in this published article.

## Abbreviations

DA: Decompression alone
DF: Decompression with fusion
ILS: Decompression with interlaminar stabilization
ISS: Decompression with interspinous stabilization
ROM: Range of motion
FE: Finite element
LSS: Lumbar spinal stenosis
